RETRACTED

# Agmatine protects retinal ganglion cells from hypoxia-induced apoptosis in transformed rat retinal ganglion cell line

**DOI:** 10.1186/1471-2202-8-81

**Published:** 2007-10-02

**Authors:** Samin Hong, Jong Eun Lee, Chan Yun Kim, Gong Je Seong

**Affiliations:** 1 Institute of Vision Research, Department of Ophthalmology, Yonsei University College of Medicine, Seoul, Korea; 2 Department of Anatomy, Yonsei University College of Medicine, Seoul, Korea

## Abstract

**Background:**

Agmatine is an endogenous polyamine formed by the decarboxylation of L-arginine. We investigated the protective effects of agmatine against hypoxia-induced apoptosis of immortalized rat retinal ganglion cells (RGC-5). RGC-5 cells were cultured in a closed hypoxic chamber (5% O_2_) with or without agmatine. Cell viability was determined by lactate dehydrogenase (LDH) assay and apoptosis was examined by annexin V and caspase-3 assays. Expression and phosphorylation of mitogen-activated protein kinases (MAPKs; JNK, ERK p44/42, and p38) and nuclear factor-kappa B (NF-κB) were investigated by Western immunoblot analysis. The effects of agmatine were compared to those of brain-derived neurotrophic factor (BDNF), a well-known protective neurotrophin for retinal ganglion cells.

**Results:**

After 48 hours of hypoxic culture, the LDH assay showed 52.3% cell loss, which was reduced to 25.6% and 30.1% when agmatine and BDNF were administered, respectively. This observed cell loss was due to apoptotic cell death, as established by annexin V and caspase-3 assays. Although total expression of MAPKs and NF-κB was not influenced by hypoxic injury, phosphorylation of these two proteins was increased. Agmatine reduced phosphorylation of JNK and NF-κB, while BDNF suppressed phosphorylation of ERK and p38.

**Conclusion:**

Our results show that agmatine has neuroprotective effects against hypoxia-induced retinal ganglion cell damage in RGC-5 cells and that its effects may act through the JNK and NF-κB signaling pathways. Our data suggest that agmatine may lead to a novel therapeutic strategy to reduce retinal ganglion cell injury related to hypoxia.

## Background

Agmatine is an endogenous polyamine that is synthesized by the decarboxylation of L-arginine by arginine decarboxylase [1,2]. It is known to be widely but unevenly distributed in the brain and other mammalian tissues [3,4]. Agmatine has been reported to have various biological actions. It stimulates the release of catecholamines from adrenal chromaffin cells [3], insulin from pancreatic islets [5], and luteinizing hormone-releasing hormone from the hypothalamus [6]. Also, it enhances analgesic effects of morphine [7], inhibits inducible nitric oxide synthase (NOS) [8], and contributes to polyamine homeostasis [2,9]. It is known that agmatine is an agonist for α2-adrenergic and imidazoline receptors [3], and an antagonist for the N-methyl-D-aspartate (NMDA) receptor [10]. However, the precise cellular mechanisms by which agmatine acts are not yet well established.

RETRACTED

Currently, a large body of experimental evidence has demonstrated the neuroprotective effects of agmatine. Agmatine reduces infarct areas and neuronal loss in cerebral ischemic and ischemic-reperfusion injury models [11-13]. It protects neurons from cell death after exposure to NMDA and glutamate [14,15]. It also attenuates the extent of neuronal loss following a spinal cord injury [16,17] and shelters neurons from glucocorticoid-induced neurotoxicity [18] and 1-methyl-4-phenyl-1,2,3,6-tetrahydropyridine-related dopaminergic toxicity [19].

On the basis of these neuroprotective effects, agmatine can be presumed to have similar neuroprotective effects on retinal ganglion cells (RGCs). Several molecules, including α2-adrenergic agonists [20-25], NMDA receptor antagonists [26-28] and NOS inhibitors [29], have been reported to protect RGCs. Agmatine also acts as an α2-adrenergic agonist [3], NMDA receptor antagonist [10], and suppressor of inducible NOS [8].

In the present investigation, we examined the protective effects of agmatine on hypoxia-induced apoptosis of RGCs by using the transformed rat RGCs (RGC-5 cell line) [30-32]. Effects of agmatine were compared to those of brain-derived neurotrophic factor (BDNF), a well-known protective neurotrophin for RGCs [33-35]. In addition, several molecular pathways associated with these neuroprotective effects of agmatine were evaluated.

## Results

### Agmatine inhibits hypoxia-induced cell damage of RGC-5 cells

We first examined the effects of hypoxia on RGC-5 cells. As shown in Figure 1, exposure to a hypoxic environment for 12, 24, and 48 hours significantly increased release of lactate dehydrogenase (LDH) by 10.17%, 20.04%, and 52.25%, respectively (all p < 0.001), thus demonstrating time-dependent hypoxia-induced neurotoxicity.

**Figure 1:** **LDH release in RGC-5 cells**. LDH release in RGC-5 cells, illustrating the neuroprotective effects of agmatine and BDNF against hypoxia for (A) 12 hours, (B) 24 hours, and (C) 48 hours. Data are shown as mean ± S.E.M. of 32 measurements. *P < 0.001.

Next, we examined the protective effects of agmatine on hypoxia-induced damage in RGC-5 cells. After 12 and 24 hours of hypoxia, agmatine treatment groups did not show significant amounts of LDH release (Fig. 1A and 1B), but there were significant effects after 48 hours of exposure (Fig. 1C). After 48 hours, the addition of 100 μM and 500 μM agmatine decreased hypoxia-induced LDH release by 25.60% and 27.09%, respectively (both p < 0.001). When the protective effects of 100 μM agmatine were compared with those of 10 ng/mL BDNF, agmatine demonstrated a more powerful protective effect than that observed for BDNF (p < 0.001).

RETRACTED

The neuroprotective effect of agmatine against hypoxia-induced damage to RGC-5 cells was further studied using Hoechst 33342 and propidium iodide (PI) double staining. The control normoxic culture exhibited confluent Hoechst-positive cells with homogeneous and compact nuclear morphology, and sparse numbers of PI-labeled cells (Fig. 2A). Exposure to hypoxia for 48 hours resulted in a significant loss of Hoechst-positive cells and many PI-positive cells with distorted and condensed nuclei (Fig. 2B). These changes were reduced by the addition of 100 μM agmatine (Fig. 2C) or 10 ng/mL BDNF (Fig. 2D) to the cultures, and agmatine had a greater protective effect.

**Figure 2:** **Hoechst 33342 and propidium iodide double staining in RGC-5 cells**. Agmatine and BDNF reduce the hypoxia-induced cell death in RGC-5. RGC-5 cells were exposed to hypoxia for 48 hours either alone (B) or in the presence of 100 μM agmatine (C) or 10 ng/mL BDNF (D). A control normoxic culture is shown in (A). The cultures were stained with Hoechst 33342 and propidium iodide. The magnification is × 400.

### Agmatine protects RGC-5 cells from hypoxia-induced apoptosis

In order to verify whether agmatine had protective effects on hypoxia-induced apoptotic death of RGC-5 cells, further analyses using annexin V assay were performed. While 12 hours of hypoxic exposure did not change the proportion of apoptotic cells compared with the normoxic culture, there were significant increases in apoptotic cells after 24 hours (Fig. 3B). With the addition of 100 μM agmatine and 10 ng/mL BDNF, the proportion of apoptotic cells decreased (Fig. 3C and 3D).

**Figure 3:** **Annexin V assay in RGC-5 cells**. Flow cytometric analysis of effects of agmatine and BDNF on the hypoxia-induced apoptosis of RGC-5 cells. Cells were exposed to hypoxia for 24 hours either alone (B) or in the presence of 100 μM agmatine (C) or 10 ng/mL BDNF (D). A control normoxic culture is shown in (A). Cultures were stained with annexin V-FITC and propidium iodide. Cells of high reactivity with FITC and low reactivity with propidium iodide (right lower area) are the apoptotic cells.

Specific caspase-3 activity was assessed using a caspase-3 assay, which could measure the cleavage of the caspase-3 specific substrate Ac-DEVD-pNA (Fig. 4). After 24 hours of hypoxic injury, the caspase-3 activity was significantly increased, and it was suppressed by 100 μM agmatine. The results obtained by adding 100 μM agmatine were similar to those seen with 50 μM caspase-3 inhibitor Z-VAD-FMK.

RETRACTED

**Figure 4:** **Caspase-3 assay in RGC-5 cells**. Colorimetric analysis of the effects of agmatine on the caspase-3 activity induced by hypoxic injury in RGC-5 cells. Cells were exposed to hypoxia for 24 hours with or without 100 μM agmatine or caspase-3 inhibitor Z-VAD-FMK (50 μM). Specific activity of caspase-3 was measured by cleavage of the caspase-3 substrate Ac-DEVD-pNA.

### Selective suppression of JNK activation by agmatine

Three mitogen-activated protein kinases (MAPKs), including c-Jun N-terminal kinase (JNK), extracellular signal-regulated kinase, (ERK) and p38 kinase (p38), were investigated using Western immunoblots. The amounts of total and phosphorylated MAPKs and β-actin are shown in Figure 5.

**Figure 5:** **Western blot analysis of MAPKs in RGC-5 cells**. Western blot analysis showing effects of agmatine and BDNF on mitogen-activated protein kinases (MAPKs). Western immunoblots probed with antibodies against JNK and phospho-JNK (A), ERK and phospho-ERK (B), p38 and phospho-p38 (C), and β-actin (D).

Total expression of the three MAPKs (JNK, ERK, and p38) and β-actin were not affected by hypoxic injury. In addition, there were no significant changes after treatment with BDNF or agmatine.

Antibodies against phospho-JNKs detected two bands at 54 and 46 kDa, and both bands had a similar tendency. Increases of phospho-JNKs in RGC-5 cells became evident 9 hours after hypoxic injury and remained elevated for 12 hours (Fig. 5A). Agmatine suppressed the hypoxia-induced phosphorylation of JNKs, but BDNF did not influence their phosphorylation.

Antibodies against phospho-ERKs also detected two bands at 44 and 42 kDa, and both bands were similar. Phospho-ERKs were not detected in the normoxic cultures. However, they were highly expressed in RGC-5 cells even after 3 hours of hypoxia and remained elevated for 12 hours (Fig. 5B). BDNF completely blocked the phosphorylation of ERKs for 6 hours, but it had no effect thereafter. In comparison, agmatine did not significantly affect the phosphorylation of ERKs.

Antibodies against phospho-p38 detected one band at 38 kDa. Phospho-p38 was not detected in normoxic cultures until 12 hours of exposure to hypoxia, but it was evident in hypoxic cultures even after 3 hours and remained elevated for 12 hours (Fig. 5C). BDNF only blocked the phosphorylation of p38 at 6 hours and agmatine had no effect on phospho-p38 levels at any time points.

Thus, phospho-MAPKs showed different activation profiles in response to hypoxic injuries in RGC-5 cells; ERK and p38 were activated relatively earlier than JNK. BDNF inhibited the activation of ERK (until 6 hours after hypoxia) and p38 (at 6 hours after hypoxia), while agmatine suppressed the activation of JNK (in significant amounts from 9 hours after hypoxia).

RETRACTED

### Suppression of NF-κB signaling by agmatine

Total expression and activation of the nuclear factor-kappa B (NF-κB) from nuclear and cytosolic fractions were evaluated separately. Representative bands from the Western immunoblots are shown in Figure 6. Antibodies against total and phospho-NF-κB bound to their respective bands at 65 kDa.

**Figure 6:** **Western blot analysis of NF-κB in RGC-5 cells**. Western blot analysis showing the effect of agmatine and BDNF on nuclear factor-kappa B (NF-κB). Western immunoblots probed with antibodies against NF-κB and phospho-NF-κB from nuclear (A) and cytosolic (B) proteins. Histone 3 (A) and β-actin (B) were used as internal controls.

In nuclear fraction, total NF-κB and histone 3 were unaffected by hypoxic injury, and there were no changes with the addition of BDNF and agmatine. However, phospho-NF-κB was significantly increased with 1 hour of hypoxia and returned to normal levels after 3 hours. This increase in phospho-NF-κB was suppressed by agmatine but not by BDNF (Fig. 6A).

In comparison, in cytoplasmic fraction, there were no significant changes in levels of phospho-NF-κB and β-actin. However, total NF-κB expression increased after 1 hour exposure to a hypoxic environment. This increase was reduced by treatment with agmatine but not BDNF (Fig. 6B).

## Discussion

Our present study demonstrates that agmatine, an endogenous polyamine with a guanidino group, prevents hypoxia-induced LDH release and apoptotic death in cultured transformed rat RGCs (RGC-5 cell line). Release of LDH was detected by LDH assay and the proportions of apoptotic cells were determined by annexin V and caspase-3 assays. Although agmatine cannot completely block cellular damage due to hypoxic injury, it has similar and even more extensive neuroprotective effects than BDNF, a well-known protective neurotrophin for RGCs [33-35]. Many molecules have been studied to rescue RGCs from glaucomatous cell death [20-29,33-35], but there is still no drug which completely shelters RGCs from injury.

In this study, undifferentiated RGC-5 cells were used instead of differentiated RGC-5 cells or primary RGCs. These immortalized cells behave differently than original RGCs, and our in vitro hypoxic model does not perfectly replicate in vivo conditions that lead to real glaucomatous injury. However, RGC-5 cells, even if they are undifferentiated, have been widely used to investigate glaucomatous RGC apoptosis as a matter of convenience [36-43]. It has been often stated that RGC-5 cells have similar characteristics to primary RGCs [30-32,44,45]. The present study using RGC-5 cells suggests a solution to the problem, although further investigations using primary cultured RGCs or in vivo glaucoma models are needed.

RETRACTED

Various functions of agmatine have been reported [3-10], but the precise cellular mechanisms of agmatine are not well established. In the present study, three types of MAPKs and NF-κB signaling pathways were evaluated. With hypoxic injury, phosphorylation of all three MAPKs and NF-κB were increased. Agmatine suppressed the hypoxia-induced activation of JNK and NF-κB, whereas BDNF inhibited the activation of ERK and p38. These differences might be caused by different mechanisms of action of the two molecules.

MAPKs are involved in highly conserved signaling pathways that regulate diverse cellular functions including cell proliferation, differentiation, migration, and apoptosis [46-48]. They are activated through phosphorylation by distinct pathways depending on stimulus and cell type. When activated, they can phosphorylate a wide range of substrates, including transcription factors and cytoskeletal proteins, resulting in specific cellular responses. In the present study, agmatine regulated the activation of JNK, but not ERK and p38, in RGC-5 cells after hypoxic injury. Our results are discrepant with those of a previous report using kidney mesangial cells under high-glucose conditions, in which agmatine was involved in the ERK pathway [49]. However, there are no reports about agmatine's effects on MAPKs in the literature, and MAPKs have been known to work differently depending on stimuli and cell types. Furthermore, due to the implications of a report demonstrating that another antagonist of the NMDA receptor MK801 can block the phosphorylation of MAPKs [50], agmatine's actions as an antagonist for the NMDA receptor [10] suggest that it might also regulate the phosphorylation of MAPKs.

In the present study, we revealed that there was an activation of NF-κB in RGC-5 cells after hypoxic injury, and agmatine was able to suppress it. Our results are consistent with previous reports that suggest that NF-κB is activated during oxidative stress [51-54]. However, Charles *et al. *[44] obtained a discrepant result in which the activity of NF-κB was decreased with serum-deprivation-induced apoptosis. While oxidative stress models, including our own hypoxic model, are based on the vascular theory of glaucoma development, the serum deprivation model is based on the mechanical pressure theory [55]. NF-κB signaling is presumed to have various responses according to the type of injury.

RETRACTED

Perhaps the most significant finding in this study was that both the increases in annexin V-positive cell number and caspase-3 activity produced by exposure of RGC-5 cells to hypoxia were counteracted by the addition of agmatine into the culture medium. This suggests that agmatine may exert a neuroprotective effect by inhibiting apoptosis in the hypoxia-injured RGC-5 cells. To our knowledge, this is the first report regarding the potential anti-apoptotic characteristics of agmatine in RGCs.

Even though this study demonstrates that activations of JNK and NF-κB were associated with the agmatine treatment, it is still not certain whether there is a close connection between neuroprotective effects of agmatine and signaling of JNK and NF-κB. However, it is presumed that they are related in some way. The ability of agmatine to regulate JNK and NF-κB pathways may contribute to protecting RGCs against hypoxia-induced cell death. Further studies are needed to elucidate the precise mechanisms by which agmatine blocks apoptosis. A deeper understanding of these mechanisms may facilitate efforts to improve the survival of RGCs from various injuries.

## Conclusion

Agmatine prevents hypoxia-induced LDH release and apoptotic death in transformed RGCs (RGC-5 cells). These neuroprotective effects of agmatine might be associated with the activity of JNK and NF-κB pathways.

## Methods

### Chemicals and antibodies

Agmatine sulfate and recombinant human BDNF were purchased from Sigma (St. Louis, MO) and R&D System, Inc. (Minneapolis, MN), respectively. Rabbit polyclonal anti-JNK p54/46, anti-ERK p44/42, anti-p38, anti-NF-κB p65, anti-phospho-JNK p54/46, anti-phospho-ERK p44/42, anti-phospho-p38, anti-phospho-NF-κB p65, and anti-histone 3 antibodies were purchased from Cell Signaling Technology, Inc (Danvers, MA). Mouse monoclonal anti-β-actin antibody was purchased from Santa Cruz Biotechnology, Inc (Santa Cruz, CA).

### Cell culture

RGC-5 cell line [30-32], a transformed RGCs developed from post-natal Sprague-Dawley rats, was grown in modified Dulbecco's modified Eagle's medium (DMEM; Gibco, Carlsbad, CA) supplemented with 10% heat-inactivated fetal bovine serum (Gibco, Carlsbad, CA) and 100 U/mL of penicillin and 100 μg/mL of streptomycin (Gibco, Carlsbad, CA). Cells were passaged every 2 to 3 days, and the cultures incubated at 37°C in 5% CO_2 _and air. During cultivation, cells exhibited the same morphological phenotype. For all experiments, cells were used at an 80% confluence.

### Hypoxic injury to retinal ganglion cells

Cultures were transferred into a closed hypoxic chamber (Forma Scientific Co., Seoul, Korea) in which oxygen level (5% O_2_, 5% CO_2_, 90% N_2_) and temperature (37°C) were automatically controlled. After washing twice with deoxygenated serum-free DMEM, cells remained in the hypoxic chamber for the designated lengths of time. Control cells were not exposed to hypoxia. Agmatine or BDNF were added to the culture medium at the start of injury as indicated.

RETRACTED

### Lactate dehydrogenase assay

Cell viability was quantified by measurement of LDH released by injured cells after hypoxic or normoxic culture for 12, 24, and 48 hours [56,57]. LDH release is expressed relative to the value of 100, which represented the maximum LDH release that occurred after freezing overnight at -70°C and subsequent rapid thawing of each culture, which induced nearly complete cell damage. All experiments were performed in at least quadruplicate and repeated at least eight times using cell cultures derived from different platings. Preliminary studies with the LDH assay tested agmatine concentrations from 10 μM to 1 mM and BDNF concentrations ranging from 5 ng/mL to 100 ng/mL. Cell death was reduced significantly at 100 μM and greater concentrations of agmatine and 10 ng/mL and greater concentrations of BDNF, so we used 100 μM agmatine and 10 ng/mL BDNF for subsequent experiments.

### Hoechst 33342 and propidium iodide staining

Apoptotic or necrotic cell death was characterized by the use of Hoechst 33342 and PI double staining [58,59]. Cells were stained with 10 μg/mL Hoechst 33342 and 10 μg/mL PI for 30 min at 37°C. After washing twice with phosphate buffered saline, cells were imaged with a digital camera attached to a fluorescence microscope.

### Annexin V assay

Percentage of cells actively undergoing apoptosis was determined by flow cytometry using the Annexin V-FITC Apoptosis Detection Kit (BD Biosciences, San Jose, CA) according to the manufacturer's instructions. Briefly, cells were harvested and resuspended in binding buffer (10^6 ^cells/mL). 10^5 ^cells were mixed with 5 μL of annexin V-FITC and 5 μL of PI. After incubating at room temperature for 15 minutes in the dark, analysis was performed by flow cytometry.

### Measurement of Caspase-3 activity

Caspase-3 activity was measured using the CaspACETM colorimetric assay system (Promega, Madison, WI) according to the manufacturer's instructions. Briefly, cells were harvested and resuspended in cell lysis buffer (10^8 ^cells/mL). After lysis, 10^6 ^cells were mixed with 32 μL of assay buffer and 2 μL of 10 mM DEVD-pNA substrate. After incubating at 37°C for 4 hours, absorbance was measured using a microplate reader at 405 nm. Absorbance of each sample was determined by subtraction of the mean absorbance of the blank from that of the sample.

RETRACTED

### Western blot analysis

For extraction of whole cellular proteins, cells were washed twice with ice-cold phosphate buffered saline and then lysed with cell lysis buffer (50 mM Tris-HCl pH 7.4, 1% NP-40, 0.25% Na-deoxycholate, 150 mM NaCl, 1 mM EDTA, 10 mM Na_3_VO_4_, 50 mM NaF, 1 mM PMSF, 1 μg/mL aprotinin, 1 μg/mL leupeptin, 1 μg/mL pepstatin) on ice for 30 minutes. Lysates were sonicated, and the cell homogenates were centrifuged at 15,000 *g *for 10 minutes (4°C).

For fractions of cytosolic and nuclear proteins, cells were lysed with lysis buffer A (10 mM HEPES pH 7.4, 10 mM KCl, 0.1 mM EDTA, 0.1 mM EGTA, 1 mM DTT, 10 mM Na_3_VO_4_, 50 mM NaF, 1 mM PMSF, 1 μg/mL aprotinin, 1 μg/mL leupeptin, 1 μg/mL pepstatin) on ice for 15 minutes, and 10% NP-40 was added. After vortexing for 10 seconds, lysates were centrifuged at 15,000 *g *for 1 minute (4°C). Supernatant was collected from the cytosolic fraction, and pellet was resuspended in lysis buffer C (20 mM HEPES pH 7.4, 400 mM NaCl, 1 mM EDTA, 1% glycerol, 1 mM DTT, 10 mM Na_3_VO_4_, 50 mM NaF, 1 mM PMSF, 1 μg/mL aprotinin, 1 μg/mL leupeptin, 1 μg/mL pepstatin) on ice for 30 minutes. Lysates were centrifuge at 15,000 *g *for 15 minutes (4°C), and supernatant was collected from the nuclear fraction.

Protein concentrations in the resultant supernatants were determined with the Bradford reagent, and equal amounts of protein (40 μg) were boiled in Laemmli sample buffer and resolved by 10 or 15% SDS-PAGE. The proteins were transferred to polyvinylidene fluoride membranes and probed overnight with antibodies against JNK, ERK p44/42, p38, NF-κB p65, phospho-JNK, phospho-ERK p44/42, phospho-p38, phospho-NF-κB, β-actin and histone 3 as indicated (diluted 1:1000). The immunoreactive bands were detected with horseradish peroxidase-conjugated secondary antibodies and visualized by enhanced chemiluminescence.

### Statistical Analysis

Data were analyzed by a two-tailed Student *t*-test or a one-way ANOVA using the Statistical Package for Social Sciences 12.0 (SPSS). Differences were considered statistically significant at p < 0.05.

## Authors' contributions

GJS and SH designed the experiments and wrote the bulk of the manuscript. SH, JEL and CYK carried out the molecular studies. All authors read and approved the final manuscript.
